RETRACTED

# Analysis of the Mechanism of Breast Metastasis Based on Image Recognition and Ultrasound Diagnosis

**DOI:** 10.1155/2021/4452500

**Published:** 2021-10-11

**Authors:** Yihong Huang, Shuo Zheng, Baoyong Lai

**Affiliations:** ^1^Fuzhou Second Hospital Affiliated to Xiamen University, Fuzhou, Fujian 350007, China; ^2^Third Affiliated Hospital of Beijing University of Chinese Medicine, Beijing 100029, China

## Abstract

Breast cancer is one of the cancers with the highest incidence among women. In the late stage, cancer cells may metastasize to a distance, causing multiple organ diseases, threatening the lives of patients. The detection of lymph node metastasis based on pathological images is a key indicator for the diagnosis and staging of breast cancer, and correct staging decisions are the prerequisite and basis for targeted treatment. At present, the detection of lymph node metastasis mainly relies on manual screening by pathologists, which is time-consuming and labor-intensive, and the diagnosis results are variable and subjective. The automatic staging method based on the panoramic image calculation of the sentinel lymph node of the breast proposed in this paper can provide a set of standardized, high-accuracy, and repeatable objective diagnosis results. However, it is very difficult to automatically detect and locate cancer metastasis areas in highly complex panoramic images of lymph nodes. This paper proposes a novel deep network training strategy based on the sliding window to train an automatic localization model of cancer metastasis area. The training strategy first trains the initial convolutional network in a small amount of data, extracts false-positive and false-negative image blocks, and uses manual screening combined with automatic network screening to reclassify the false-positive blocks to improve the class of negative categories. Using mammography, ultrasound, MRI, and 18F-FDG PET-CT examinations, the detection rate and diagnostic accuracy of primary cancers in the breast of patients with axillary lymph node metastasis as the first diagnosis were obtained. The detection rate and diagnostic accuracy of breast MRI for primary cancers in the breast are much higher than those of X-ray, ultrasound, and 18F-FDG PET-CT (all *P* values <0.001). Mammography, ultrasound, and PET-CT examinations showed no difference in the detection rate and diagnostic accuracy of primary cancers in the breast of patients with axillary lymph node metastasis as the first diagnosis. Breast MRI should be used as a routine examination for patients with axillary lymph node metastasis as the first diagnosis. The primary breast cancer in the first diagnosed patients with axillary lymph node metastasis is often presented as localized asymmetric compactness or calcification on X-ray; it often appears as small focal mass lesions and ductal lesions without three-dimensional space-occupying effect on ultrasound.

RETRACTED

## 1. Introduction

Breast cancer is a common malignant tumor that threatens women's lives. Breast-conserving surgery can be performed when detected early, and the prognosis is good, and the five-year survival rate is high. However, radical resection may be necessary after the middle and late stages; not only the quality of life is significantly reduced, but the 5-year disease-free survival rate is also significantly reduced, which increases the economic burden of patients [1, 2]. Early detection of lesions is critical. Commonly used methods of breast cancer diagnosis include mammography, ultrasound, and magnetic resonance imaging [3]. As a classic breast cancer screening method, molybdenum target has a high penetration rate at home and abroad, especially abroad. It is very sensitive to intralesional calcification, and it is highly sensitive to the diagnosis of tumors with calcification, especially for nonmass cancers with calcification, and the detection rate is significantly higher than that of ultrasound [4]. However, for noncalcified masses, the detection rate is affected by the compactness of the breast glands. At the same time, its radioactivity limits the age and frequency of screening. MRI has high definition and high resolution. MRI enhancement has a high sensitivity for the diagnosis of breast cancer. This has been recognized. The sensitivity of the diagnosis of breast cancer reaches 95%–99%. MRI also has many functional imaging methods. For example, diffusion-weighted imaging, magnetic resonance power, magnetic resonance perfusion imaging, etc., can increase the description of the internal biological characteristics of the tumor on the basis of morphology and provide help for the diagnosis of early breast cancer [5]. However, MRI cannot be used as a screening method due to its high scanning cost [6].

In order to increase the accuracy of breast cancer diagnosis and reduce the missed diagnosis rate, it is urgent to combine tumor internal functional imaging on the basis of morphology to assist diagnosis. Malignant tumor cells generate a large number of capillaries in the early stage of formation. Tumor cells are metabolized and consume a large amount of oxygen in the blood, resulting in a state of rich blood supply and hypoxia inside the tumor, resulting in a significant increase in intravascular hemoglobin, especially deoxyhemoglobin [7, 8]. The changes in the internal metabolic function of these malignant tumors are obviously different from those of benign tumors. Ultrasonic Light Scattering Imaging System (DOT) combines ultrasound imaging technology and photon scattering tomography technology. You can use ultrasound to locate the suspicious area, emit near-infrared light through the probe, and use hemoglobin and deoxyhemoglobin as the main absorbers of near-infrared light to measure total hemoglobin, which indirectly reflects the distribution of blood vessels and oxygen and state in the tissue, thereby providing tissue deficiency [9]. Ultrasonic light scattering imaging system realizes the scanning of tumor internal metabolic function on the basis of morphology. At present, there are more researches focusing on injecting the tumor surface or areola skin with ultrasound contrast agent, tracking the movement of lymph vessels to find the sentinel lymph node in the armpit, and then performing the contrast and biopsy of the sentinel lymph node to confirm whether it has metastasis. However, the procedure is complicated and it is a traumatic test. How to predict the metastasis of axillary lymph nodes under the premise of simplicity and non-invasiveness is a challenge [10].

RETRACTED

This paper proposes a method based on deep convolutional neural network that can automatically locate and identify the cancer metastasis area in the panoramic image of breast lymph nodes. Specifically, the technical contributions of this article can be summarized as follows:

1. Through targeted data expansion and training strategies, the cancer metastasis recognition model of the image block is obtained. Then, the model is sent to the preprocessed panoramic image, and the predicted calorific value map about the probability of cancer metastasis is obtained. The model proposed in this paper can better identify cancer metastasis areas and greatly reduce false positive areas, and the model has higher sensitivity.
2. We retrospectively analyzed axillary tumors in a cancer hospital from January 2018 to November 2020, with axillary tumors as the first diagnosis, and performed breast MRI examination. The axillary tumor was confirmed to be lymph node metastatic adenocarcinoma by biopsy, and the results of immunohistochemical examination supported the original disease. The lesions came from breast tissue, and no obvious malignant lesions were found on clinical palpation of bilateral breasts in 73 patients. Among them, 61 cases underwent mammography at the same time, 69 underwent breast ultrasound at the same time, 19 underwent MRI-guided “second-eye” ultrasound examination, and 22 underwent 18F-FDG PET-CT at the same time.
3. Two senior breast imaging diagnosticians analyzed the X-ray images, ultrasound images, and MRI images of all cases, and evaluated the composition of breast tissue according to the breast imaging report and data system standards proposed by the American College of Radiology. This topic aims to analyze the mammography, ultrasound, MRI, and 18F-FDG PET-CT manifestations of patients with axillary lymph node metastasis cancer as the first diagnosis (negative breast clinical palpation), and to compare the effects of different imaging methods in the primary breast. The diagnosis efficiency of cancer foci provides a basis for the clinical development of diagnosis and treatment plans.

RETRACTED

## 2. Related Work

Rac1 and Cdc42 are generally believed to promote the invasion and metastasis of breast cancer [11]. However, the relationship between Rho A and breast cancer metastasis remains controversial. The traditional view is that the expression level of Rho A is positively correlated with the pathological stage of breast cancer and the degree of lymph node metastasis, and based on this, it is believed that Rho A can promote the migration and invasion of tumor cells [12]. However, related scholars have constructed a breast cancer cell line that stably interferes with Rho A and found that the invasion ability of this cell is significantly enhanced [13]. It is speculated that Rho A can hinder the invasion of breast cancer cells. These two diametrically opposed views indicate that the relevant mechanisms still need to be studied in depth.

Extracellular signal regulated kinase (ERK) is a key regulatory molecule that transmits signals from cell surface receptors to the nucleus [14]. The RAS/ERK signaling pathway plays an important role in the occurrence and development of breast cancer and other epithelial tumors. Studies have shown that SHP2 participates in the RAS/ERK signaling pathway and plays an important regulatory role [15]. In the study of lung cancer and cartilage tumors, it was found that through the stimulation of EGF, IL-6, and other growth factors or cytokines, the phosphatase domain of SHP2 can activate the RAS signaling pathway and phosphorylate SHP2 after autophosphorylation [16]. Phosphorylated SHP2 dephosphorylates and inactivates the inhibitory proteins in the RAS/ERK pathway such as SHPS-1 and palmitoyl phosphoprotein Sprouty, thereby lifting the inhibitory state of the RAS/ERK pathway. They found that SHP2 can continuously activate the RAS/ERK signaling pathway by activating Src Family Kinases (SFKs) [17].

The p LKO.1-puro vector is a lentiviral sh RNA expression vector, which can efficiently and stably infect mammalian cells. Puromycin can be used to screen mutant cell lines. In this experiment, in order to obtain a stable O-Glc NAc expression inhibiting breast cancer cell model, they used the p LKO.1-puro vector to construct an OGT-specific interference vector, which effectively detected the OGT expression in breast cancer cells 4T1 [18].

RETRACTED

Studies have shown that PUGNAc can efficiently and specifically inhibit the activity of OGA in vivo and in vitro, thereby increasing the level of O-Glc NAc in cells [19]. In this experiment, a breast cancer cell model with elevated O-Glc NAc was obtained by PUGNAc treatment [20]. In order to ensure the reliability of subsequent experiments, in most experiments, they used both OGT silencing and PUGNAc treatment of two cell models [21]. A large number of studies have shown that the absence or excessive expression of O-Glc NAc can lead to cell cycle inhibition and apoptosis [22]. At the same time, considering the expression of O-Glc NAc in normal breast cells, this article did not completely inhibit the expression of OGT and the activity of OGA in order to study the role of O-Glc NAc in the occurrence and development of breast cancer.

In addition, because tumor metastasis is an overall process, animal experiments should be considered to prove the effect of Gankyrin on tumor metastasis from the overall level. At present, the animal models of breast tumor metastasis are relatively mature. Commonly used are breast fat pad injection model and tail vein injection model. In addition to the observation and counting of metastases by naked eyes, the analysis methods include in vivo imaging analysis and pathological section analysis. The relevant animal experiments of Gankyrin's effect on breast cancer metastasis are being actively prepared [23]. Preliminary preparations are to construct a mouse breast cancer metastasis model through breast fat pad injection and to observe the degree of metastasis through animal in vivo fluorescence imaging technology [24]. Through transfection and screening, breast cancer cells stably expressing luciferase have been obtained.

In another liver cancer study, it was also found that SHP2 can effectively promote the activation of ERK [25]. The activated ERK can significantly inhibit the activity of B lymphocyte tumor-2 protein, thereby inhibiting cell apoptosis and leading to cell cancerization. In the related research of Noonan syndrome, related scholars found through mouse model experiments that inhibiting the protein expression of SHP2 can significantly inhibit the phosphorylation of ERK, and the abnormal activation of SHP2 can overactivate the phosphorylation of ERK1/2 [26]. At present, the role of SHP2 in the RAS/ERK signaling pathway of breast cancer cells remains to be further clarified. Relevant scholars have selected breast cancer cell lines MDA-MB-231 cells and BT549 cells as the research objects, by constructing recombinant plasmids (shSHP2-NC1, shSHP2-NC3) that reduce the expression of SHP2 stably and small interfering RNA fragments that reduce the expression of SHP2 transiently (SiSHP2-1#, siSHP2-2#), analyzing the effect of downregulation of SHP2 protein level on ERK signaling pathway. The experimental results show that in MDA-MB-231 and BT549 cells, the steady decrease or transient decrease of SHP2 protein level will cause the phosphorylation level of ERK to decrease significantly [27]. This indicates that in breast cancer cells, SHP2 participates in the RAS/ERK signaling pathway and plays a positive regulatory role.

RETRACTED

## 3. Research Methods

### 3.1. Inspection Method

We instruct the patient to take a supine position, hold the head with both hands, and fully expose both breasts and armpits. First, we use a two-dimensional probe to perform routine scans on both breasts and axilla. After the tumor is found, we select the largest section of the lesion and the section with the most abundant blood flow (try to show part of the surrounding glandular tissue as a control) and keep the probe position and patient position unchanged, adjust various machine parameters. During the imaging process, the patient is instructed to maintain the position, avoid deep breathing, and the operator to avoid overpressurization of the probe and maintain the stability of the probe. The storage time is at least 3 minutes. After the contrast is completed, the dynamic images stored in the machine are played back. Two sonographers (mammography work ≥5 years) will analyze the enhanced features. If there is a disagreement, another senior ultrasound is required. The physician participates in the analysis and finally reaches a consistent diagnosis opinion. The specific process of inspection is shown in Figure 1.

### 3.2. Histological Grade and Immunohistochemical Determination

Experienced pathologists will diagnose the submitted specimens. For the determination of the expression of ER, PR, HER-2, and Ki-67, we used the SP staining method. If the tumor cell nuclear staining is greater than or equal to 10%, it is judged to be positive for ER and PR; if the tumor cell nuclear staining is less than 10%, it is judged to be negative for ER and PR. We judged the nucleus brown staining ≥14% as Ki-67 positive, and the brown-yellow staining nucleus less than 14% as negative. After HER-2 is stained with SP, the cell membrane with brown particles appears as the number of stained positive cells ≥10% as +, the number of stained positive cells ≥20% is considered to be 2+, and the number of stained positive cells ≥30% is considered to be 3+. Among them, “−” or “+” is judged as negative, “+++” is judged as positive, and “++” is judged as positive by HER-2 gene amplification, and if there is gene amplification, it is judged as positive, and if there is no gene amplification, it is judged as negative.

RETRACTED

Histopathological grading used Scarff–Bloom–Richardson grading system to divide invasive ductal carcinoma into grade I (highly differentiated), grade II (moderately differentiated), and grade III (poorly differentiated), and axillary lymph node metastasis was recorded.

### 3.3. Analysis Method

We refer to the relevant content of the breast imaging report data system BI-RADS to understand the patient's menstrual cycle, and compare and observe the bilateral breasts, pay attention to the two-dimensional characteristics of the tumor and the color Doppler data for quantitative analysis. For lesion cases, it is necessary to focus on analyzing the differences in sonograms between the lesions to find out the similarities and differences; whether there are catheters connected between the lesions, if catheter lesions are found, we scan the long and short axis of the catheter to observe whether there is any inside the catheter expansion, echo, and presence or absence of solid nodules; if there are nodules, we observe the morphological boundary and the presence or absence of blood flow; for some solid tumors in the breast, the elastic image can be analyzed to understand its softness and hardness. The ultrasound classification of small breast cancer is divided into 5 types, as shown in Table 1.

We use SPSS 23.0 statistical analysis software. The features of breast cancer enhanced ultrasound imaging include enhancement level, enhancement method, filling defect, range change, and perforating vessels. The correlation analysis of tumor size, axillary lymph node metastasis, histopathological grade, immunohistochemical index ER, PR, HER-2, and Ki-67 expression was analyzed by Pearson's chi-square test and Fisher's exact probability method.

## 4. Automatic Segmentation Model of the Breast Lymph Node Cancer Metastasis Area

### 4.1. Image Preprocessing of the Metastatic Area of Breast Lymph Node Cancer

The digitized panoramic image is huge in size and has many white background areas. In order to reduce the calculation time, this article first preprocesses the panoramic image to remove non-histopathological areas to reduce the computational complexity of the digitized pathological image. Panoramic images are usually stored in a multiresolution pyramid structure, containing multiple downsampled samples of the original image, and the image with the largest resolution is called level 0, and the other versions from bottom to top are called level 1 and level 2; the image size of each level differs by approximately 2 times. In order to reduce the amount of calculation in the white unorganized area, this paper uses a multilevel mapping strategy based on the pyramid structure to exclude the unorganized area.

RETRACTED

The focus of the pyramid structure multilevel mapping strategy lies in coordinate mapping. Through a specific threshold method, the coordinates of the tissue area are obtained under the low-resolution image, and then the coordinates are mapped to the high-resolution according to the pyramid structure. This paper chooses the image at the 7th level of the pyramid structure as the input image of the coordinate mapping and then obtains the coordinates of the tissue area under the low-resolution image through a specific image algorithm.

The flowchart of removing the background in low-resolution images is shown in Figure 2. First, the image is grayed out, and then two binary images are obtained using the maximum difference between classes method, and then the two binary images are merged according to the AND operation, and the white area obtained is the region of interest containing the tissue area. In this paper, we use a closed operation with a disc structure of 3 × 3 pixels to reduce the omission of the tissue area, and an open operation with a disc structure of 8 × 8 pixels to remove small impurity areas, and the final result is an image focusing only on the organized area.

In the pyramid structure of the panoramic image, one pixel at level 4 resolution is equivalent to an image block with a size of 256 × 256 pixels under level 0 resolution image. Therefore, when the pixels at the level 4 resolution only slide in the organized area, the sliding window with the size of 256 × 256 pixels at the corresponding position under the level 0 resolution image also slides only in the organized area, as shown in Figure 3.

We establish the image grayscale histogram and normalize the grayscale histogram. Suppose the original gray level *N*, the number of pixels with gray level *i* is *n*_*i*_, and calculate the probability of the appearance of pixels with gray level *p*_*i*_:

(1) $$\begin{array}{c} p_{i}=\frac{n_{i}}{\left|\prod_{i=1}^{L}n_{i-1}\right|}. \end{array}$$

Assuming that *A* represents the background (gray level is 0∼*N*) and *B* represents the target, for the two types of pixels *A* and *B*, the probability of each category is

(2) $$\begin{array}{c} P_{A}=\prod_{i=1}^{t+1}\left(P_{i}\cdot P_{i+1}\right),\\ P_{B}=\prod_{i=t+2}^{L}\left(P_{i}\cdot P_{i+1}\cdot P_{i+2}\right). \end{array}$$

Finally, we calculate the between-class variance of the two regions, *A* and *B*:

(3) $$\begin{array}{c} w_{A}=\prod_{i=1}^{t+1}\left(iP_{A}P\right),\\ w_{B}=\prod_{i=1}^{L}\left(iP_{B}P_{i+1}\right),\\ w_{0}=\prod_{i=1}^{L}i\left(p_{A}w_{A}-p_{B}w_{B}\right),\\ \sigma^{2}=0.5p_{A}{\left(w_{0}-w_{A}\right)}^{2}-0.5p_{B}{\left(w_{0}-w_{B}\right)}^{2}. \end{array}$$

Among them, *w*_*A*_ and *w*_*B*_ are the average gray values of the *A* and *B* regions, respectively; *w*_0_ is the global gray average of the gray image; and *σ*^2^ is the between-class variance of the *A* and *B* regions. The algorithm calculates the optimal threshold to maximize the distinction between the tissue area and the white background area in the pathological image.

RETRACTED

### 4.2. Deep Learning Model Based on the Sliding Window

The construction of training set is the key to network training. This paper first randomly extracts hundreds of thousands of image blocks with a sliding window of 256 × 256 pixels. If the center of these blocks is within the cancer metastasis area marked by the pathologist, they are positive blocks and marked as 0; otherwise, they are negative blocks. As the AlexNet model converges quickly during training, this article chooses to use AlexNet as the initial network and further extracts the training set based on the initial prediction results. First, an initial binary classification model is trained based on AlexNet and applied to the prediction of the panoramic image of the training sample, so as to obtain an initial segmentation probability map about cancer metastasis.

We extract a large number of image blocks of false positive and false negative regions and recombine them to obtain millions of positive and negative image blocks. Due to the imbalance in the number of samples of positive and negative blocks and the high probability of false positives, this paper reclassifies the negative blocks in the training set to expand the difference between classes and facilitate the model to better identify positive and negative. It is finally classified into 5 categories. Except for the positive category, the other 4 categories are all negative categories, and are marked as negative category 1, category 2, and category 3 according to the characteristics of the block such as more blanks, more cells, and normal black. For negative blocks that are very similar to positives, they are marked as category 4, which is called similar positive category. In addition, in order to reduce the workload of manually selecting data, this article uses a special training strategy to select data and train the model. Considering the calculation cost and calculation time, this article does not use Inception, ResNet, DenseNet, and other networks, but uses VGG-16 with moderate parameters and calculation time as the final five-class network. In order to improve the robustness of the model, in addition to data enhancement such as rotation and mirroring of image blocks, this paper also adds a data enhancement method for H&E dye transformation, which can imitate the color change caused by the proportion of H&E dye reagent. The calculation steps are as follows:

First, we convert the extracted image block from color (RGB) space to optical density (OD) space:

(4) $$\begin{array}{c} \text{OD}=-2\;\log_{10}\left(0.12I\right). \end{array}$$

Then, we delete the OD sensitivity of less than 0.12 and create a plane by performing singular-value decomposition on the processed OD value and taking the eigenvectors corresponding to the two largest eigenvalues:

(5) $$\begin{array}{c} \text{OD}⇄VS⟶V^{-1}\left|\text{OD}\right|, \end{array}$$

where *I* is the color space of the image; OD is the optical density space; and *V* and *S* are the corresponding coloring vectors.

RETRACTED

## 5. Results and Analysis

### 5.1. Pathologically Confirmed Ultrasound Findings of Primary Breast Lesions

Sixty-nine patients underwent breast ultrasound examination, of which 60 underwent radical mastectomy and 9 underwent breast-conserving surgery. Pathological examination results showed that 56 cases were breast cancer, and 13 cases were not found to be cancerous. Among the 60 patients who underwent radical mastectomy, 59 underwent radical mastectomy for axillary masses on the ipsilateral side, and 1 case underwent contralateral radical mastectomy for axillary masses on the opposite side of the breast due to MRI findings. Among 56 patients with breast cancer confirmed pathologically, 15 patients (26.8%) had breast cancer lesions detected by ultrasound examination of the breast, of which 10 patients (66.7%) showed hypoechoic masses, and 2 patients (13.3%) showed breast cancers. There were many hypoechoic areas along the catheter, 2 cases (13.3%) showed hypoechoic areas along the catheter, and 1 case (6.7%) had catheter dilation with intra-catheter calcification. The diameter of the mass was 0.5 cm∼1.7 cm; 8 cases showed irregular shape, 2 cases were round or oval, 9 cases had unclear borders, and 1 case had clear borders. The blood flow in 6 cases was not abundant, the blood flow in 3 cases was rich, and the blood flow in 1 case was marginal; 5 cases had no rear acoustic shadow, 4 cases had increased rear echo, and 1 case had increased rear echo.

41 cases of primary breast cancer were not detected by ultrasound, of which 39 cases were detected by breast MRI, 23 cases were nonlumps, and 16 cases were tumors, as shown in Figure 4. The diameter of the mass was 0.67 cm∼1.56 cm; 10 cases showed irregular shape, 6 cases were oval or round, with irregular edges; after multiphase dynamic enhancement, the inside of the lesion showed uneven enhancement in 12 cases and uniform enhancement in 3 cases. The enhancement distribution of nonmass lesions included 10 cases of linear enhancement, 7 cases of segmental enhancement, 5 cases of focal enhancement, and 1 case of multiple regional enhancement; 16 cases of uneven enhancement, 4 cases of uniform enhancement. There were 3 cases of ring enhancement; 13 cases of type I (increasing type) TIC, 5 cases of type II (platform type), and 5 cases of type III (outflow type).

RETRACTED

Among 39 patients, 19 cases underwent MRI-guided “second-eye” ultrasound examination, 10 cases (52.6%) showed hypoechoic masses, and 5 cases (26.3%) showed localized hypoechoic areas. It showed that there were multiple hypoechoic areas distributed along the catheter, and 1 case (5.3%) showed that the catheter was dilated and the interior was hypoechoic. The diameter of the mass was 0.6 cm∼2.0 cm, with an average of (1.1 ± 0.4) cm; the masses were all irregular, with unclear borders; 5 cases of masses had inadequate blood flow; and 3 cases of masses had abundant blood flow. There were 2 cases of mass marginal blood flow; 7 cases had no posterior acoustic shadow; 2 cases had posterior acoustic shadow and 1 case had posterior echo enhancement; 2 cases had hypoechoic masses with calcification; and 1 case had ductal dilation. 5 cases of primary breast cancer showed a localized hypoechoic area. The tumors with this appearance did not have a three-dimensional space-occupying effect. Corresponding to their MRI findings, 3 cases showed focal enhancement and 2 cases showed linear enhancement. Three cases of primary breast cancer showed multiple hypoechoic areas along the duct. Corresponding to their MRI findings, 2 cases showed segmental enhancement and 1 case showed linear enhancement.

Among the 60 patients with breast cancer confirmed pathologically, 58 patients had primary breast cancers detected by MRI. The analysis of FGT of 58 cases of breast showed that 36 cases of breast fibroadenoid tissues were unevenly distributed, 16 cases were scattered fibroadenous tissues of breast, and 4 cases were extremely dense. At the same time, after multiphase dynamic enhancement, the mammary fibroglandular background showed slight enhancement in 45 cases, mild enhancement in 11 cases, and moderate enhancement in 2 cases.

The 58 cases of cancer foci detected by MRI included 38 cases of nonmass lesions and 20 cases of mass lesions. The diameter of the mass was 0.7 cm∼1.7 cm; 12 cases showed irregular shape, 8 cases were oval or round, with irregular edges; after multiphase dynamic enhancement, the inside of the lesion showed uneven enhancement in 13 cases and uniform enhancement in 4 cases. The distribution of enhancement of nonmass lesions includes 14 cases of linear enhancement, 13 cases of segmental enhancement, 9 cases of focal enhancement, and 2 cases of multiple regional enhancement; there are 25 cases of uneven enhancement, 8 cases of uniform enhancement, and clusters within the lesion. There were 4 cases of shape enhancement and 1 case of clustered small ring enhancement; 16 cases of TIC were type III (outflow type), 15 cases were type I (increasing type), and 7 cases were type II. The MRI appearance of the primary breast lesion is shown in Figure 5.

RETRACTED

Two cases of primary cancer in the breast were not detected by MRI. One patient was diagnosed with a left axillary mass as the first patient and underwent radical mastectomy on the left side. DCIS components were found outside the left breast through whole breast specimens and were found in the left breast. Retrospective analysis of the MRI image of this patient showed that the fibroglandular tissues of the affected breast showed uneven distribution. After dynamic enhancement, the fibroglandular background showed moderate enhancement, and there were many spots distributed along the ducts. Another patient was first diagnosed with a left axillary mass and underwent radical mastectomy on the left side. A nonspecial invasive carcinoma with a maximum diameter of 2 mm was found on the upper left side of the left breast through the whole breast. A retrospective analysis of the patient's MRI image showed that the fibroglandular tissues of the affected breast showed uneven distribution. After dynamic enhancement, the fibroglandular background showed moderate enhancement, with multiple patches and enhancements along the duct.

### 5.2. X-Ray Findings of Primary Breast Lesions Confirmed by Pathology

Sixty-one patients underwent mammography, of which 53 underwent radical mastectomy and 8 underwent breast-conserving surgery. Pathological examination results showed that 51 cases were breast cancer, and 10 cases were not found to be cancerous. Of the 53 patients who underwent radical mastectomy, 51 underwent radical mastectomy for axillary masses on the ipsilateral side, and 2 cases underwent contralateral radical mastectomy due to suspicious tumors in the contralateral breast of the axillary mass on MRI. Among 51 cases of breast cancer confirmed pathologically, 16 cases of breast cancer were detected by breast X examination. Analysis of the composition of the breast tissues of 16 patients showed that 9 cases of mammary glands were scattered with fibrous glands, and 7 cases of mammary glands were uneven and dense. The primary cancers in the breast detected by X-ray examination showed 8 cases of simple localized asymmetry and compactness, 5 cases of simple calcification, 1 case of simple mass (the mass was irregular, edge burr, and high density), and the mass was accompanied by calcification. From the morphology of calcification, 3 cases showed fine polymorphic calcification, 2 cases showed amorphous calcification, and from the distribution of calcification, 2 cases showed regional distribution, and 2 cases showed calcification. Cases were distributed in segments, and 1 case was distributed in clusters.

RETRACTED

X-rays of primary cancers in 35 cases of breast cancer were not detected. Among them, 15 cases showed uneven and dense breasts, 12 cases showed scattered fibrous glands, 5 cases were almost all adipose tissue, and 3 cases were extremely dense. Among these 35 breast cancer patients, 33 cases were examined by breast MRI to detect primary cancers in the breast, of which 22 cases showed no masses and 11 cases showed masses. The diameter of the mass was 0.72 cm∼1.61 cm; 8 cases showed irregular shape, 4 cases were oval or round, with irregular edges; after multiphase dynamic enhancement, the inside of the lesion showed uneven enhancement in 8 cases and uniform enhancement in 3 cases. There was 1 case with clusters of small ring enhancement; 7 cases of type II (platform type), 4 cases of type III (outflow type), and 1 case of type I (increasing type) TIC. The enhancement distribution of nonmass lesions included 8 cases of focal enhancement, 7 cases of linear enhancement, and 6 cases of segmental enhancement. There were 11 cases of type I (increasing type), 6 cases of type III (outflow type), and 4 cases of type II (platform type). The MRI findings of primary cancers in the breast that were not detected by mammography are shown in Figure 6.

### 5.3. 18F-FDG PET-CT Findings of Primary Breast Lesions Confirmed Pathologically

22 patients underwent 18F-FDG PET-CT examination. 19 cases underwent radical mastectomy for axillary tumors on the ipsilateral side, and 3 cases underwent breast-conserving surgery. Pathological examination results showed that 19 cases were breast cancer, and 3 cases were not found to be cancerous. Among the 19 cases of breast cancer confirmed pathologically, 5 cases of breast cancer were detected by 18F-FDG PET-CT, all of which were mass lesions, and the diameter of the tumor was 1.1 cm∼1.6 cm.

14 cases of primary breast cancer were not detected by 18F-FDG PET-CT, 13 cases of which were detected by breast MRI examination, including 8 cases of nonmass lesions and 5 cases of mass lesions. The diameter of 5 cases was 0.8 cm∼1.2 cm, of which 3 cases were less than 1.0 cm. The enhancement distribution of nonmass lesions included 6 cases of linear enhancement, 1 case of segmental enhancement, and 1 case of focal enhancement.  Table 2 shows the MRI findings of cancers in the breast that were not detected by 18F-FDG PET-CT. Mammography, ultrasound, MRI, and 18F-FDG PET-CT examinations for clinically palpable axillary lymph node metastases in patients with axillary lymph node metastases are shown in Figures 7 and 8, respectively.

RETRACTED

## 6. Conclusion

The degree of lymph node metastasis is one of the important criteria for determining the pathological staging of breast cancer. Early detection and early diagnosis are the key to the treatment of breast cancer. In the image analysis module of the breast cancer lymph node metastasis staging system, the deep learning method is used to automatically locate and identify the cancer metastasis area in the panoramic image of the breast lymph node. And the accuracy of the model has reached a relatively high level, which can support the feature extraction and selection work. Of the 73 patients, 63 underwent radical mastectomy, 9 underwent breast-conserving surgery, and 1 underwent MRI-guided “second-eye” ultrasound-guided puncture. Pathologically confirmed 60 cases of breast cancer, including 41 cases of nonspecific invasive carcinoma, 9 cases of ductal carcinoma in situ, 2 cases of invasive micropapillary carcinoma, and 2 cases of invasive lobular carcinoma. There were 2 cases of microinvasive carcinoma, and 1 case of glycogen-rich clear cell carcinoma. No cancer was found in the specimens of 11 cases of radical breast surgery and 2 cases of breast-conserving surgery. The detection rate and diagnostic accuracy of breast MRI examinations for primary cancers in the breast are significantly higher than those of X-ray, ultrasound, and 18F-FDG PET-CT examinations. There is no difference in the detection rate and diagnostic accuracy of primary cancers. MRI examination of the breast should be used as a routine examination for patients with axillary lymph node metastasis as the first diagnosis. Primary breast cancer in patients with axillary lymph node metastasis as the first diagnosed patient often showed localized asymmetric compactness or calcification on X-ray; it often showed small focal mass lesions and ductal lesions without three-dimensional space-occupying effect on ultrasound. MRI often presents as small focal mass lesions and linear, segmental, or focal nonmassive lesions with enhanced distribution; 18F-FDG PET-CT often presents as a mass lesion with a diameter >1.0 cm.

RETRACTED

## Figures and Tables

**Figure 1:** The specific process of breast metastasis examination.

**Figure 2:** Image removal background flowchart. (a) Top view of the panoramic image. (b) Grayscale. (c) Binary image after special threshold processing. (d) Binary image with closed operation. (e) Binary image with open operation. (f) The nonblack area is the tissue area that needs to be calculated.

**Figure 3:** Panoramic scan image structure and multilevel mapping strategy.

**Figure 4:** MRI appearance of breast cancer not detected by breast ultrasound. MRI findings of primary breast lesions confirmed by pathology.

**Figure 5:** MRI appearances of primary breast lesions. (a) Mass morphology. (b) Internal enhancement characteristics of the tumor. (c) Tumor time-signal intensity curve type. (d) Nonmass distribution. (e) Nonmass internal enhancement features. (f) Nonlump time-signal intensity curve type.

**Figure 6:** MRI findings of primary cancers in the breast that were not detected by mammography.

**Figure 7:** Detection rate of MRI, X-ray, ultrasound, and 18F-FDG PET-CT.

**Figure 8:** Diagnostic accuracy rate of MRI, X-ray, ultrasound, and 18F-FDG PET-CT.

**Table 1:** Ultrasound classification of small breast cancer.

Type	Feature
Nodular type	Nodules with the largest diameter of the lesion ≦1 cm
Mass type	The maximum diameter of the lesion >1 cm, ≦2 cm; according to the boundary of the lesion, it can be divided into the following: Type I (clear boundary type): the boundary of the lesion is clear, but there is no obvious envelope; Type II (rough edge type): the edge of the lesion is blurred, showing small burr-like shape, partly with angle sign
Capsule type	The lesion was a mixed nodule with cysts and solids
Catheter type	The catheter is tortuous and dilated, and the lesions are distributed along the inner wall of the dilated catheter
Diffuse type	The lesion showed a hypoechoic area with unclear borders and no obvious nodular echo

**Table 2:** MRI findings of breast cancers not detected by 18F-FDG PET-CT.

Breast tissue composition on MRI	Nonlumps	Lumps
Fibroglandular tissue is scattered	1	2
Slight enhancement of fibroglandular background	1	12
Almost entirely composed of adipose tissue	1	0
Moderate enhancement of fibroglandular background	0	1
Fibroglandular tissue is unevenly distributed	5	4

## Data Availability

The data used to support the findings of this study are available from the corresponding author upon request.

## References

[1] O’Loughlin D., O’Halloran M., Glavin M., Jones E., Moloney M., Elahi M. A. (2018). Microwave breast imaging: clinical advances and remaining challenges. *IEEE Transactions on Biomedical Engineering*.

RETRACTED

[2] Wang R., Li J., Zhao Y., Li Y., Yin L. (2018). Investigating the therapeutic potential and mechanism of curcumin in breast cancer based on RNA sequencing and bioinformatics analysis. *Breast Cancer*.

[3] Porter E., Coates M., Popovic M. (2016). An early clinical study of time-domain microwave radar for breast health monitoring. *IEEE Transactions on Biomedical Engineering*.

[4] Sparano J. A., Gray R. J., Makower D. F. (2015). Prospective validation of a 21-gene expression assay in breast cancer. *New England Journal of Medicine*.

[5] Rodrigues R., Braz R., Pereira M., Moutinho J., Pinheiro A. M. G. (2015). A two-step segmentation method for breast ultrasound masses based on multi-resolution analysis. *Ultrasound in Medicine and Biology*.

[6] Miglioretti D. L., Lange J., van den Broek J. J. (2016). Radiation-induced breast cancer incidence and mortality from digital mammography screening. *Annals of Internal Medicine*.

[7] Song H. E. A. (2017). Detectability of breast tumor by a hand-held impulse-radar detector: performance evaluation and pilot clinical study. *Scientific Reports*.

[8] Jafari S. H., Saadatpour Z., Salmaninejad A. (2018). Breast cancer diagnosis: imaging techniques and biochemical markers. *Journal of Cellular Physiology*.

[9] Modiri A., Goudreau S., Rahimi A., Kiasaleh K. (2017). Review of breast screening: toward clinical realization of microwave imaging. *Medical Physics*.

[10] Park K., Chen W., Chekmareva M. A., Foran D. J., Desai J. P. (2017). Electromechanical coupling factor of breast tissue as a biomarker for breast cancer. *IEEE Transactions on Biomedical Engineering*.

[11] Morais P., Queiros S., Meester P. D. (2018). Fast segmentation of the left atrial appendage in 3-D transesophageal echocardiographic images. *IEEE Transactions on Ultrasonics, Ferroelectrics, and Frequency Control*.

[12] Casu M. R., Vacca M., Tobon J. A. (2017). A COTS-based microwave imaging system for breast-cancer detection. *IEEE Transactions on Biomedical Circuits and Systems*.

[13] Di Meo S., Svelto F., Summers P. E. (2017). On the feasibility of breast cancer imaging systems at millimeter-waves frequencies. *IEEE Transactions on Microwave Theory and Techniques*.

[14] Tuminello S., Liu B., Wolf A., Alpert N., Taioli E., Flores R. M. (2018). Comparison of in-hospital and long-term outcomes of sublobar lung cancer surgery by VATS and open techniques. *American Journal of Clinical Oncology*.

[15] Sasada S., Masumoto N., Goda N. (2018). Which type of breast cancers is undetectable on ring-type dedicated breast PET?. *Clinical Imaging*.

[16] Reis S., Gazinska P., Hipwell J. H. (2017). Automated classification of breast cancer stroma maturity from histological images. *IEEE Transactions on Biomedical Engineering*.

RETRACTED

[17] Hu Y., Guo Y., Wang Y. (2019). Automatic tumor segmentation in breast ultrasound images using a dilated fully convolutional network combined with an active contour model. *Medical Physics*.

[18] Pandya H. J., Park K., Chen W., Goodell L. A., Foran D. J., Desai J. P. (2016). Toward a portable cancer diagnostic tool using a disposable MEMS-based biochip. *IEEE Transactions on Biomedical Engineering*.

[19] Martellosio A., Bellomi M., Pasian M. (2017). Dielectric properties characterization from 0.5 to 50 GHz of breast cancer tissues. *IEEE Transactions on Microwave Theory and Techniques*.

[20] Jensen M.-B., Nielsen T. O., Knoop A. S., Laenkholm A.-V., Balslev E., Ejlertsen B. (2018). Mortality and recurrence rates among systemically untreated high risk breast cancer patients included in the DBCG 77 trials. *Acta Oncologica*.

[21] Turkki R., Byckhov D., Lundin M. (2019). Breast cancer outcome prediction with tumour tissue images and machine learning. *Breast Cancer Research and Treatment*.

[22] Badrinarayanan V., Kendall A., Cipolla R. (2017). SegNet: a deep convolutional encoder-decoder architecture for image segmentation. *IEEE Transactions on Pattern Analysis and Machine Intelligence*.

[23] Kumar S., Srinivasan A., Nikolajeff F. (2018). Role of infrared spectroscopy and imaging in cancer diagnosis. *Current Medicinal Chemistry*.

[24] Palumbo C., Cyr S.-J., Mazzone E. (2019). Impact of tumor size on cancer-specific mortality rate after local tumor ablation in T1a renal-cell carcinoma. *Journal of Endourology*.

[25] Bonnefoi H., Grellety T., Tredan O. (2016). A phase II trial of abiraterone acetate plus prednisone in patients with triple-negative androgen receptor positive locally advanced or metastatic breast cancer (UCBG 12-1). *Annals of Oncology*.

[26] Traina T. A., Miller K., Yardley D. A. (2018). Enzalutamide for the treatment of androgen receptor-expressing triple-negative breast cancer. *Journal of Clinical Oncology*.

[27] Poompavai S., Gowri Sree V. (2018). Dielectric property measurement of breast-tumor phantom model under pulsed electric field treatment. *IEEE Transactions on Radiation and Plasma Medical Sciences*.

